RETRACTED

# Antihypertensive Activity in High Salt-Induced Hypertensive Rats and LC-MS/MS-Based Phytochemical Profiling of *Melia azedarach* L. (Meliaceae) Leaves

**DOI:** 10.1155/2022/2791874

**Published:** 2022-07-26

**Authors:** Anam Saeed, Kashif Bashir, Abdul Jabbar Shah, Rahila Qayyum, Taous Khan

**Affiliations:** ^1^Department of Pharmacy, COMSATS University Islamabad, Abbottabad Campus, Abbottabad 22060, Pakistan; ^2^Gomal Medical College, MTI, Dera Ismail Khan, KPK, Pakistan

## Abstract

*Melia azedarach* L. leaves have been traditionally used but not scientifically evaluated for antihypertensive activity. The focus of the present work was to carry out the detailed phytochemical profiling and antihypertensive potential of methanolic extract and subsequent fractions of this plant. The tandem mass spectrometry-based phytochemical profiling of *M. azedarach* extract (Ma.Cr) and fractions was determined in negative ionization mode while molecular networking was executed using the Global Natural Product Social (GNPS) molecular networking platform. This study resulted in the identification of 29 compounds including flavonoid *O*-glycosides, simple flavonoids, triterpenoidal saponins, and cardenolides as the major constituents. Ma.Cr at the concentration of 300 mg/kg resulted in a fall in blood pressure (BP), i.e., 81.44 ± 2.1 mmHg in high salt-induced hypertensive rats *in vivo*, in comparison to normotensive group, i.e., 65.36 ± 1.8 mmHg at the same dose. A decrease in blood pressure was observed in anaesthetized normotensive and hypertensive rats treated with extract and various fractions of *M. azedarach*. A reasonable activity was observed for all fractions except the aqueous fraction. The highest efficacy was shown by the ethyl acetate fraction, i.e., 77.06 ± 3.77 mmHg in normotensive and 88.96 ± 1.3 mmHg in hypertensive anaesthetized rats. Ma.Cr and fractions showed comparatively better efficacy towards hypertensive rats as compared to rats with normal blood pressure. Blood pressure-lowering effects did not change upon prior incubation with atropine. *In vitro* testing of Ma.Cr and polarity-based fractions resulted in _L_-NAME sensitive, endothelium-dependent vasodilator effects on aortic tissues. Pretreatment of aorta preparations with Ma.Cr and its fractions also blocked K^+^-induced precontractions indicating Ca^2+^ channel blocking activity comparable to verapamil. The extract and polarity-based fractions did not reveal a vasoconstrictor response in spontaneously beating isolated rat aorta. Ma.Cr and fractions when used in atrial preparations resulted in negative inotropic and chronotropic effects. These effects in atrial preparations did not change in the presence of atropine. These effects of extract and fractions explained the antihypertensive potential of *M. azedarach* and thus provided a scientific basis for its ethnopharmacological use in the treatment of hypertension. Among the constituents observed, flavonoids and flavonoid *O*-glycosides were previously reported for antihypertensive potential.

RETRACTED

## 1. Introduction

Hypertension is one of the serious medical conditions that dramatically increases the probability of different health-related issues [1]. It is a noncommunicable global disease with lack of initial symptoms and a high mortality rate and is termed a silent killer. Approximately, 1.13 billion people around the world are suffering from hypertension, including the majority of people from countries with low and middle income [2]. The overall prevalence of hypertension in Pakistan was 26.34% (25.93%, 26.75%) [3]. Currently, several drugs are used for the treatment of hypertension such as calcium channel blockers, *β*-blockers, ACE inhibitors, and diuretics [4, 5]. Treatment of hypertension requires a combination of drugs that are acting at various therapeutic sites and thus result in adverse effects. These adverse effects need further management that leads to complications in the treatment of hypertension. Alternatively, herbal drugs that possess a therapeutically important combination of constituents have various clinical issues [6]; therefore, research is being carried out to find out more effective remedies with lesser side effects.

Natural products obtained from plants have been major contributors to the drug discovery against various diseases. A large population of Asia relies on local remedies for the treatment of different diseases including cardiovascular disorders [7, 8]. Research has confirmed the cardiovascular activity of many plant constituents like allicin from *Allium sativum*, digoxin from *Digitalis purpurea*, curcumin from *Curcuma longa*, and tetrandrine from *Stephania tetrandra* [9, 10].

*M. azedarach* L. (Meliaceae) is one of the plants used by community practitioners for the treatment of hypertension [11]. It is commonly known as Chinaberry or China tree in English and dharek or darek in Urdu [12]. Traditionally, it is used for the management of inflammation, cardiovascular disorders, and leprosy [13, 14] and also as a diuretic, astringent, and wormicidal [15], whereas its oil is used in cramps and rheumatism [16]. It is applied in the Ayurvedic and Unani medicinal system as an analgesic, antioxidative, rodenticidal, and insecticidal and also to treat diabetes, diarrhea, and hypertension [12]. It contains several groups of phytoconstituents like steroids, flavonoids, acids, and terpenoids [12]. The constituents previously reported from this plant include quercetin, kaempferol (flavonoids), campesterol, stigmasterol (phytosterols), phytol (diterpene), heptadecane, *β*-sitosterol, hexadecanoic acid, tocopherol, *β*-carotene, 1-eicosanol (triterpene), terpene alcohol and squalene [17], *β*-D-glucopyranose, daucosterol, liminoid glycoside, melianol, meliacarpin, meliacin, (±) pinoresinol, and hydroxyl-3-methoxycinnamaldehyde and terpenoids such as azadirachtin-A and azadirachtin-B [18].

RETRACTED

*M. azedarach* leaf extracts possess antiviral [19] and antifertility [20] activities, while fruit extract possesses ovicidal [21], larvicidal [22], and antioxidant activity [13, 23]. Its aqueous extract possesses reducing agent potential [24]. It is reported to have antidiabetic potential by inhibiting the effects of the protein tyrosine phosphatase enzyme [25]. Green synthesis of silver nanoparticles of methanolic crude extract of the plant was carried out, which showed antimicrobial, antibacterial, antidiabetic, and wound healing activities [26–28]. Anticancer activity on MCF-7 cell lines was reported on methanolic extract of *M. azedarach* [29]. Studies suggest that phenolics and phytosterols from this plant are important for cosmetics and pharmaceutical applications [30]. Consequently, current studies were undertaken to investigate the antihypertensive potential and vasorelaxant effects of *M. azedarach* and to provide scientific support for the traditional claim of curing hypertension. Furthermore, the constituents in bioactive fractions were dereplicated using LC-MS/MS-based GNPS molecular networking to identify chemical space.

## 2. Methods

### 2.1. Chemicals

Phenylephrine hydrochloride (PE) (S2569), atropine sulfate (CFN90575), acetylcholine chloride (Ach) (CFN90038), norepinephrine (NE) (CFN90047), N*_*ω*_*-nitro L-arginine methyl ester hydrochloride (_L_-NAME) (CFN60352), and potassium chloride (104938) were procured from Sigma-Aldrich (US). Injection pentothal sodium was purchased from Abbott Laboratories (Pakistan) whereas injection heparin was purchased from F. Hoffmann-La Roche (Switzerland), respectively.

### 2.2. Extraction of Plant Material

Leaves of *M. azedarach* were collected from Dera Ismail Khan, Khyber Pakhtunkhwa, Pakistan, in the month of July. The leaf specimen was authenticated by Dr. Abdul Nazir, Associate Professor, Department of Environmental Sciences, COMSATS University Islamabad, Abbottabad Campus, Pakistan, and the sample voucher (Ma.L.05/17) was deposited. The leaves were washed, garbled, and dried in shade followed by pulverization to fine particles. The extract was prepared by macerating about 18 kg of the powdered plant material in methanol at ambient temperature, i.e., 23-25°C for 3 weeks, 1 week, and 3 days, respectively, with random stirring [31]. The filtrate was obtained by passing through qualitative grade 1 filter paper (Whatman filter paper). The extract was prepared by concentrating under vacuum using a rotary evaporator. Further polarity-based fractions of the extract were prepared including *n*-hexane (18 g), ethyl acetate (4 g), chloroform (26 g), *n*-butanol (16 g), and aqueous fraction (30 g) using previously reported method [31].

RETRACTED

### 2.3. LC-MS/MS-Based Phytochemical Analysis

Phytochemical profiling of the extract and fractions was determined using Orbitrap Velos Pro mass spectrometer (Thermo Fisher Scientific, Germany). The detector used in the chromatographic system was a photodiode array (PDA) detector. The samples were ionized using the ESI technique in negative ionization mode. The solvent system used was prepared using formic acid 0.1% in water (A) and 0.1% formic acid in acetonitrile (B) and was run in the gradient fashion. The gradient elution program was set as the concentration of B for 0.5 min was 5%; for 0.5-6.5 min, B was 5-95%; for 6.5-8.5 min, B was 95%; and for 8.5-10 min, B was 95-5%. The volume of the sample injected was 10 *μ*L at the flow rate of 0.5 mL/min. At the *m*/*z* range of 110-2000, spectra were recorded. The LC-MS/MS data were collected and interpreted with help of the Thermo Xcalibur software. The LC-MS/MS data, which included parameters like retention time, MS-MS fragmentation pattern, *m*/*z*, dereplication results, and molecular formula. GNPS molecular networking platform was used for phytochemical profiling of the *M. azedarach* extract and fractions. MS convert package from the ProteoWizard software was used to convert all mass spectrometry data into GNPS compatible “.mzxML” format. WinSCP, a recommended FTP client, was used for uploading the files on the GNPS platform. Various features of the spectral data were made visible with the help of Cytoscape 3.8.2. For identification of the majority of metabolites present, MolNetEnhancer tool was used. The outcomes of GNPS analysis were thoroughly compared with the outcome of manual interpretation [32].

### 2.4. Pharmacological Studies

#### 2.4.1. Experimental Animals and Housing Conditions

Sprague-Dawley (SD) rats, preferably male, in the weight range of 200-220 g were acquired and kept at the animal house of the university. The temperature was maintained between 23 and 25°C. The protocol was carried out according to the Institute of Laboratory Animal Resources Commission on Life Sciences, National Research Council [33], and endorsed by the Ethical Committee of CUI, Abbottabad Campus, in a meeting called on 7-09-2021 vide approval no. PHM-Eth/CS-M02-060-0721.

RETRACTED

#### 2.4.2. Invasive Blood Pressure Recording

Both normotensive and hypertensive rats were used for this study, and the protocol as previously described [34] was used with some modifications. SD rats, preferably male, were housed in a hygienic environment and fed on 8% sodium chloride (NaCl, Scharlau, Spain) in food and water for 8 weeks. Sodium thiopental, 50-90 mg/kg intraperitoneally, was used to induce anaesthesia in rats. Polyethylene tubing (PE-20) was used for cannulation in order to help animal respire spontaneously, whereas polyethylene tubing (PE-50) was used to cannulate right carotid artery, attached to pressure transducer hyphenated to bridge amplifier and PowerLab Data Acquisition System (AD Instruments, Australia). In order to facilitate the injection of standards, Ma.Cr, and fractions, left jugular vein was cannulated. After a stabilization period of 20 min, the animal was injected with 0.1 mL saline or a test sample. Then, after a waiting period of 10-15 min when the arterial blood pressure was stabilized, standards and test materials were injected intravenously after that a flush of 0.1 mL saline was given. The effects of standards such as Ach (1 *μ*g/kg) and NE (1 *μ*g/kg) were monitored before injecting test material. Hypertensive rats with a BP of 150-190 mmHg were used for the study [35, 36].

#### 2.4.3. Safety Studies

Balb-C mice weighing 20-25 g were used in the study for safety tests [37, 38]. These were arranged into four groups (*n* = 5). Increasing doses of plant extract, i.e., 1 g/kg, 3 g/kg, and 5 g/kg, were fed to the animals in 10 mL/kg of saline serving as trial groups. To one group, saline was given (10 mL/kg, p.o.) and was considered as negative control group. During a 24 h test period, the mice were monitored for mortality and toxic symptoms such as anorexia, diarrhea, and lethargy.

### 2.5. *In Vitro* Experiments

#### 2.5.1. Vascular Reactivity Studies

From both normal and hypertensive SD rats, thoracic aortic tissue was carefully removed and placed in Kreb's solution. It was then prepared by cutting into 3 mm rings and hung in an organ bath in the presence of Kreb's solution and carbogen (5 percent carbon dioxide in oxygen). The organ bath was hyphenated to force transducer and PowerLab Data Acquisition System (AD Instruments, Australia). By changing buffer after every 15 min, the tissue was set to stabilize (60-90 min) at 2 g resting tension. Endothelium was intentionally damaged in a few aortic rings. To check endothelium integrity, after stabilization, contractions were induced with PE (1 *μ*M) that were inhibited using Ach (1 *μ*M). For 20-30 min, aortic ring preparations were incubated using _L_-NAME (10 *μ*M). The vasorelaxation produced by the extract and fractions was monitored in the absence as well as in presence of _L_-NAME. Responses to the test samples were tested in parallel in denuded tissues and tissues of hypertensive rats [36, 39].

RETRACTED

#### 2.5.2. Isolated Right Atrial Preparations

SD rats were used to check how the rate and force of contraction were affected by extract and fractions in right atrial preparations [40]. After dissection of the animal, the right atria was taken out and hung in a 10 mL organ bath filled with Kreb's solution at 32°C and in the presence of carbogen connected to a pressure transducer, which was hyphenated with a PowerLab Data Acquisition System. Pacemaker activity of atria caused it to beat freely during the equilibrium period (30 min) at preload of 1 g. Some tissues were incubated with atropine (1 *μ*M) to check if muscarinic receptor activation was involved.

### 2.6. Statistical Analysis

The mean standard error (±SEM) was used to express the data from the animal and *in vitro* investigations. The statistical differences between the treatments and the control were assessed using the IBM SPSS software and ANOVA followed by Tukey's test (version 20, SPSS Inc., Chicago, IL). Significance was determined at ∗*p* < 0.05, ∗∗*p* < 0.01, and ∗∗∗*p* < 0.001.

## 3. Results

### 3.1. Metabolomic Results and Dereplication

In the current study, spectroscopic analysis and GNPS molecular networking were used to study the complete phytochemical profile of the extract and polarity-based fractions of *M. azedarach* leaves. Twenty nine compounds in total were determined in the Ma.Cr and fractions. The major constituents observed belonged to flavonoid *O*-glycoside, triterpenoids, lipids, and saponins.  Table 1 enlists the compounds tentatively identified in the Ma.Cr and fractions in negative ion mode showing their retention time, MS/MS fragmentation patterns, and *m*/*z* values. *n*-Hexane fraction showed the presence of isoquercetin, kaempferol 7-*O*-hexosyl(1-2) deoxyhexoside, soyacerebroside-I, quercetin 3-*O*-neohesperidoside, fatty acid 18 : 4, monogalactosyl monoglycerol, and digalactosyl monoglycerol. The cluster containing quercetin 3-*O*-alpha-L-[6^‴^-p-coumaroyl-beta-D-glucopyranosyl-(1->2)-rhamnopyranoside] and quercetin-3-*O*-[2-*O*-6-*z*-*p*-coumaroyl-glucopyranoside]-rhamnopyranoside was observed separately as shown in Figure 1. Triterpenoidal glycosides like cardenolides, momordicoside, and genistin were observed in Ma.Cr, chloroform fraction, and *n*-hexane fraction, respectively, as shown in Figure 2. The observed constituents in chloroform fraction included kaempferol-7-*O*-neohesperidoside, quercetin, quercetin-3-*O*-[2-*O*-6-z-*p*-coumaroyl-glucopyranoside]-rhamnopyranoside, soyacerebroside I, keracyanin, isosakuranetin-7-*O*-neohesperidoside, and momordicoside. Constituents observed in the ethyl acetate fraction consisted of kaempferol 3-*O*-[2-*O*-(glucopyranoside)]-rhamnopyranoside, quercetin, and isoquercetin. Furthermore, isoquercitrin, isorhamnetin-3-*O*-galactoside-6^″^-rhamnoside, kaempferol 3-*O*-robinoside-7-*O*-rhamnoside, 7-*O*-methyl genistein, quercetin 3-*O*-[2^″^-*O*-(6^‴^-*O*-*p*-coumaroyl)-*β*-D-glucopyranosyl]-*α*-L-rhamnopyranoside, rutin, sulfobacin B, and nicotiflorin were tentatively detected in *n*-butanol fraction. In aqueous fraction, quercetin 3-*O*-[2-*O*-6-*Z*-*p*-coumaroyl-glucopyranoside]-rhamnopyranoside and quercetin 3-*O*-(2^″^-*O*-glucopyranoside)-rhamnopyranoside were observed. Flavonoid *O*-glycosides are grouped in one cluster (purple coloured) as shown by molecular networking analysis (Figure 1). The fragmentation of flavonoid *O*-glycosides as seen in a representative UV-chromatogram, total ion chromatogram, and mass spectra is given in Figures 3–5.

RETRACTED

### 3.2. Pharmacological Studies

#### 3.2.1. Safety Studies

The Ma.Cr in the concentration of 1, 3, and 5 g/kg was determined to be safe in mice, with no evidence of lethality after 24 h of observation along with no behavioral changes, anorexia, diarrhea, or lethargy.

#### 3.2.2. Antihypertensive Effect

Standards like NE (1 *μ*M) and Ach (1 *μ*M) were given before the administration of Ma.Cr and fractions. These drugs induced an increase and a decrease in blood pressure, respectively (Figure 6(a)). Blood pressure in normotensive and high blood pressure animals was 118 ± 4.13 (*n* = 15) and 160 ± 3.22 (*n* = 15), respectively. Ma.Cr was intravenously administered to the normotensive group after anesthetization, which resulted a fall in mean arterial pressure (MAP). At the dose levels of 1, 3, 10, 30, 100, 150, and 300 mg/kg of Ma.Cr, a concentration-dependent lowering of MAP, i.e., 2.53 ± 1.6, 8.36 ± 1.3, 15.43 ± 2.7, 26.23 ± 2.1, 37.82 ± 1.2, 51.85 ± 1.1, and 65.36 ± 1.8 mmHg, was observed, respectively (Figure 6(c)). All fractions tested reduced MAP, with the ethyl acetate fraction at 300 mg/kg dose showing the highest efficacy (77.06 ± 3.77) (Figure 7(a)). When compared to pretreated groups, the percent decrease in all cases was statistically significant (*p* ≤ 0.05) at different doses as shown in Figures 7(a)–7(e). Prior incubation of the tissue with atropine (1 *μ*M) did not change the effects produced with Ma.Cr and fractions (data not shown).

RETRACTED

#### 3.2.3. Antihypertensive Effect on Hypertensive Rats

Ma.Cr caused a significant decrease in MAP in hypertensive rats under anaesthesia than in the normotensive groups. By the administration of Ma.Cr, the % decrease in MAP at dose levels of 1, 3, 10, 30, 100, 150, and 300 mg/kg was 3.51 ± 2.8, 8.95 ± 3.2, 15.6 ± 3.5, 28.49 ± 4.3, 57.4 ± 5, 73.71 ± 3.0, and 81.44 ± 2.1 mmHg (Figure 6(c)). Ethyl acetate fraction had the highest blood pressure-lowering effect when compared with other fractions. It caused a percent fall in MAP of 5.44 ± 1.6, 13.66 ± 1.8, 24.00 ± 4.4, 34.78 ± 4.8, 50.77 ± 5.2, 77.41 ± 3.02, and 88.96 ± 1.3 mmHg, at respective doses (Figures 7(a)–7(e)). Atropine (1 *μ*M) pretreatment did not alter the responses produced by Ma.Cr and fractions (data not shown).

#### 3.2.4. Nitric Oxide Release-Dependent Effect

The response of Ma.Cr and fractions was determined using the tissues that induced more than 80% relaxation upon administration of acetylcholine. The contractions were induced with phenylephrine (PE) (1 *μ*M) in rings with intact endothelium. The addition of Ma.Cr in the cumulative pattern caused nitric oxide (NO) release-based vasorelaxation showing the EC_50_ of 0.70 mg/mL (0.5–1.2). _L_-NAME incubation of intact tissue resulted in an inhibition of the vasorelaxation potential of Ma.Cr, and only 20% relaxation was observed (Figure 8(b)). Ma.Cr did not significantly relax the denuded tissue even at increasing doses. It only induced 26% relaxation at the highest dose. Ma.Cr did not relax the tissue in hypertensive rats' aorta rings precontracted with PE and elicited only 37% relaxation. Similar results were obtained with ethyl acetate fraction on rat aorta. Endothelium-dependent vasorelaxation was elicited in intact tissue with the EC_50_ value of 0.086 mg/mL (0.05-0.13). The vasorelaxant effect was blocked in intact tissues upon incubation with _L_-NAME (10 *μ*M), tissues with damaged endothelium and hypertensive groups. Chloroform, *n*-hexane, and *n*-butanol like crude extract also elicited NO release-dependent relaxation (Figures 8(b)–8(g)). The blood pressure-lowering effect produced by Ma.Cr and its fractions was unaffected upon treatment of tissue with atropine (1 *μ*M) (data not shown).

High K^+^ (80 mM) was utilized to see if the crude extract and fractions have any effect on vascular smooth muscles. Relaxation was caused by the addition of different concentrations of extract and fractions in a cumulative pattern (Figure 9(a)). High efficacy was observed with the ethyl acetate fraction whereas the aqueous fraction has lower activity and caused only partial inhibition. A typical calcium channel blocker, verapamil, was used to induce the endothelium-independent relaxant effect as shown in Figure 9(b).

RETRACTED

#### 3.2.5. Studies on Atrial Tissues

Rhythmic contractions and relaxations were exhibited by right atria from normotensive animals where the use of acetylcholine in cumulative pattern blocked force (negative inotropic) and rate (negative chronotropic) of contraction, which was also blocked with atropine thus confirming the protocol (Figure 10(a)). The crude extract caused partial inhibition of both rate and force of atrial contractions with the EC_50_ of 4.18 mg/mL (3.9-8.08) and 5.29 mg/mL (4.71-10.0), respectively. The ethyl acetate fraction completely blocked both rate and force of atrial contractions with the EC_50_ of 1.38 mg/mL (0.3-1.68) and 0.75 mg/mL (0.55-1.30), respectively (Figure 10(b)). Atropine incubation did not alter either of these responses.

Rate and force of atrial contractions were fully inhibited in the presence of *n*-hexane fraction showing the EC_50_ of 2.34 mg/mL (1.66-4.0) and 1.95 mg/mL (0.9-2.85), respectively. On the other hand, the chloroform, *n*-butanol, and aqueous fraction did not induce suppression (Figures 10(c)–10(f)). Preincubation with atropine did not alter the responses of these fractions as well.

## 4. Discussion

The methanolic extract of leaves of *M. azedarach* was phytochemically analyzed using LC-MS/MS and GNPS molecular networking. The outcomes of phytochemical profiling showed 29 compounds including simple flavonoids, flavonoid *O*-glycosides, glycoglycerols, fatty acids, and glycerophosphoinositols, which are varied in terms of structure and fragmentation patterns. Glucose, rhamnose, and pentose were observed, respectively, at 162, 146, and 132 Da as a result of fragmentation of flavonoid-*O*-glycosides [41]. Previously, quercetin, rutin, isoquercetin, kaempferol 7-*O*-neohesperidoside, isorhamnetin 3 *O*-rutinoside, and isosakuranetin 7-*O*-neohesperidoside were reported from *M. azedarach* using LC-MS/MS analysis [42]. One metabolite is representing each node in molecular networking analysis, marked based on its *m*/*z* value. On the basis of similarity in their core chemical structure and fragmentation pattern, different metabolites are grouped accordingly. The ethyl acetate fraction with highest potential as an antihypertensive consisted of the flavonoid *O*-glycosides, i.e., isoquercetin and kaempferol 3-*O*-[2-*O*-(glucopyranoside)] rhamnopyranoside. By the fragmentation of isoquercetin and rutin, quercetin was obtained whereas isorhmnetin-3-*O*-rutinoside and isorhmentin-3-*O*-glucoside were fragmented to give isorhamnetin. The *n*-hexane fraction contained flavonoid glycosides along with phospholipids and exhibited higher activity after ethyl acetate. The molecular networks of flavonoid *O*-glycosides observed in *M. azedarach* are shown in Figure 1.

RETRACTED

Safety studies of the plant were carried out to determine the safety profile for oral use at different doses. It was found that the plant is safe for up to 5 g/kg oral dose. Using an invasive blood pressure approach, Ma.Cr and fractions have a relaxant effect in both normotensive and hypertensive anaesthetized rats, being more potent in hypertensive rats, indicating its antihypertensive potential. The ethyl acetate fraction had a greater relaxant effect when Ma.Cr and fractions were compared. Similarly, in high salt-induced hypertensives rats, the ethyl acetate fraction was found to be more effective. BP is the multiple of cardiac output and peripheral resistance [43, 44]. On the basis of the above-mentioned outputs, this plant was considered for further study *in vitro* to determine the underlying blood pressure-lowering mechanism.

Ma.Cr and ethyl acetate fractions relaxed PE (1 *μ*M) induced precontraction in an isolated tissue with an intact endothelium, suggesting the possible involvement of nitric oxide (NO-endothelium-derived relaxing factor) [45]. NO is a powerful vasodilator produced by NO synthase in the endothelium [46] and causes vascular relaxation [47]. Ma.Cr and its fractions did not show a relaxation response to PE (1 *μ*M) in high salt-induced hypertensive rat aorta even at higher doses. It has been shown that high dietary salt decreases plasma nitrate and impairs endothelial function [36, 48]. Inhibition of NO synthase or increased superoxide production may be responsible for the unavailability of NO-dependent vascular relaxation [49]. When the tissue was pretreated with _L_-NAME, an inhibitor of nitric oxide synthase [50, 51], it reduced the vasorelaxant effect caused by Ma.Cr and fractions similar to denuded tissues. This is an evidence of the involvement of endothelium-based relaxation and NO release.

Ma.Cr and fractions were studied on PE (1 *μ*M) and high K^+^ (80 mM) based contractions in aortic tissue to determine their effect on voltage-dependent calcium channels (VDCs) [52]. Mechanism of high K^+^ (80 mM) induced contractions involves vascular smooth muscle cells and the opening of voltage-dependent L-type Ca^++^ channels, as a result of which extracellular Ca^++^ enters the cells and produces contractions [36]. The substance that blocks these contractions is recognized as the blocker of Ca^++^ influx [53]. When added cumulatively to the precontracted aortic ring, the Ma.Cr and fractions were more potent against PE (1 *μ*M) in comparison to high K^+^-induced contractions (80 mM) [54].

RETRACTED

The release of calcium from internal stores and also from receptor-operated calcium channels (ROCs) was considered to be blocked by Ma.Cr and its fractions as a result of relaxation of PE (1 *μ*M) contractions. Ma.Cr and its fractions were found to be devoid of any contraction upon cumulative addition to the steady-state baseline.

The atrial preparations were studied to determine the involvement of cardiac function in antihypertensive activity. The rate and force of atrial contraction were completely suppressed when atrial preparations were treated with Ma.Cr, ethyl acetate, and *n*-hexane fraction. However, the aqueous, *n*-butanol, and chloroform fractions did not show similar results. Pretreatment of atrial tissues with atropine was carried out to rule out possible involvement of cardiac muscarinic receptor activation in effect of Ma.Cr and fractions. As a result, it was found that rate and force of atrial contraction were not affected by this pretreatment, and thus, muscarinic receptors are not involved [36]. From these results, it can be assumed that decrease in rate and force of atrial contraction may also be related to blockade of calcium transport, i.e., its release from internal stores or influx through VDCs.

The phytochemical profiling demonstrated the richness of the extract and fractions in flavonoid glycosides. Previous studies have shown that flavonoid glycosides contribute to cardiovascular protection [55, 56] and possess anticholinesterase activity [57]. For that reason, the flavonoids present in this plant may be responsible for antihypertensive activity. Similarly, it has been reported that quercetin, kaempferol (flavonoids), campesterol, and stigmasterol (phytosterols) are the key chemical constituents of *M. azedarach* extract [17]. Quercetin, an anticholinesterase [58] and antihypertensive [59] constituent, may be involved in the fall in MAP.

Based on the phenolic profile, we speculate that the antihypertensive activity of *M. azedarach* extract may be partly related to its flavonoid contents. Ma.Cr and its fraction possess vasorelaxation effects through nitric oxide pathways and maybe through calcium channel blocking. Plant-based constituents have vasodilator potential through multiple pathways like NO pathways [60] or through inhibition of calcium release from Ca^++^ stores [45] in addition to many other mechanisms.

## 5. Conclusion

Detailed phytochemical studies of *M. azedarach* leaves were carried out by highly sensitive LC-MS/MS technique and GNPS molecular networking. Flavonoid *O*-glycosides, terpenoidal saponins, terpenoidal glycosides, and simple flavonoids were tentatively determined in *M. azedarach* leaves. Flavonoid glycosides were considered to be a major constituent in Ma.Cr and bioactive fractions. Current findings on the cardiovascular activities of *M*. *azedarach* extract and fractions revealed that it contains phytoconstituents that mediate the relaxant effect via the NO pathway, which could explain its antihypertensive effect. These findings provide a pharmacological foundation for *M. azedarach*'s traditional medical use as an antihypertensive remedy.

RETRACTED

## Figures and Tables

**Figure 1:** Molecular networking analysis of *M. azedarach* leaf extract showing presence of flavonoid *O*-glycosides using tandem mass data in negative ion mode.

**Figure 2:** GNPS molecular networking outcomes of tandem mass analysis of *M. azedarach* crude extract indicating the presence of terpenoidal glycosides.

**Figure 3:** UHPLC-PDA-MS/MS analysis of crude extract from *M. azedarach* leaves in negative ion mode. UHPLC-PDA chromatogram of crude extract (a) and total ion chromatogram in negative ion mode (b).

**Figure 4:** UHPLC-PDA-MS/MS analysis of *n*-butanol fraction from *M. azedarach* leaves in negative ion mode. UHPLC-PDA chromatogram of *n*-butanol fraction (a) and total ion chromatogram in negative ion mode (b).

**Figure 5:** MS2 fragmentation pattern of quercetin 3-*O*-neohesperidoside (rutin) *m*/*z* is 609.15 (MS1) (a) and MS2 fragmentation pattern of kaempferol 7-*O*-neohesperidoside *m*/*z* is 593.15 (MS1) (b) from *M. azedarach* leaf extract.

**Figure 6:** The hypertensive and hypotensive effects of norepinephrine (NE) and acetylcholine (ACh), respectively. (a) The blood pressure of normotensive and hypertensive rats. (b) The effect of crude extract of *M. azedarach* (Ma.Cr) (c) on MAP in normotensive and hypertensive rats, under anesthesia (*n* = 6-7); ^∗^*p* < 0.05, ^∗∗^*p* < 0.01, and ^∗∗∗^*p* < 0.001.

**Figure 7:** Graphs show the effect of ethyl acetate (Ma.EtOAc) (a), *n*-hexane (Ma.*n*-Hex) (b), chloroform (Ma.Chl) (c), *n*-butanol (Ma.*n*-but) (d), and aqueous (Ma.Aq) (e) fractions of *M. azedarach* on mean arterial pressure (MAP) in normotensive and hypertensive rats, under anesthesia. Values shown are mean ± SEM (*n* = 6 − 7); ^∗^*p* < 0.05, ^∗∗^*p* < 0.01, and ^∗∗∗^*p* < 0.001.

**Figure 8:** Graphs show the response of acetylcholine (a), crude extract of *M. azedarach* (Ma.Cr) (b), its fractions ethyl acetate (Ma.EtOAc) (c), *n*-hexane (Ma.*n*-Hex) (d), chloroform (Ma.Chl) (e), *n*-butanol (Ma.*n*-But) (f), and aqueous (Ma.Aq) (g) on PE-induced contractions in intact (with and without _L_-NAME (10 *μ*M) pretreatment), denuded aortic rings from normotensive rats and rings from hypertensive rats. Values shown are mean ± SEM (*n* = 6-7); ^∗^*p* < 0.05, ^∗∗^*p* < 0.01, and ^∗∗∗^*p* < 0.001.

RETRACTED

**Figure 9:** Graph shows vasodilator effect of crude extract of *M. azedarach* (Ma.Cr), its fractions ethyl acetate (Ma.EtAc), n-Hexane (Ma.nHex), chloroform (Ma.Chl), n-butanol (Ma.n-but) and aqueous (Ma.Aq) (a) verapamil (b) on high K^+^ (80 mM)-induced contractions in isolated rat aorta rings. Values shown are mean ± SEM (*n* = 6-7); ^∗^*p* < 0.05, ^∗∗^*p* < 0.01, and ^∗∗∗^*p* < 0.001.

**Figure 10:** Concentration-response curves show the effect of crude extract (Ma.Cr) (a), and fractions, i.e., *n*-hexane (Ma.*n*-hexane) (b), chloroform (Ma.Chl) (c), ethyl acetate (Ma.EtOAc) (d), *n*-butanol (Ma.*n*-but) (e), and aqueous (Ma.Aq) (f) of *M. azedarach* on spontaneously occurring rate and force of contraction in isolated SD rat right atrial preparations. The values shown are mean ± SEM (*n* = 5).

**Table 1:** Phytochemical profile of *M. azedarach* leaf extract and fractions using tandem mass analysis.

Compound No.	Rt	[M-H]^−^m/z	MS2 fragmentation ion [M-H]^−^	Dereplication results	Exact Mass (g/mol)	Molecular Formula
Crude extract of *M. azedarach* leaves						

1	4.80	395.11	377.72, 374.95, 348.68 (100), 312.58	3,4',5,6,7-pentamethoxyflavone	372.12	C_20_H_20_O_7_
2	5.22	341.10	322.96 (100), 320.64, 300.58	(8,8 dimethyl-2,10-dioxo-9H- pyrano [2,3-f] chromen-9-yl)(*Z*)-2-methylbut-2-enoate	342.11	C_19_H_18_O_6_
3	5.96	449.22	426.83, 377.78, 232.47, 222.48, 151.831 (100)	Strophanthidine	404.21	C_23_H_32_O_6_
4	4.06	464.38	442.84, 432.77, 414.85, 342.58, 298.31(100)	Isoquercetin	464.09	C_21_H_20_O_12_
5	4.06	623.16	623.80, 605.66, 590.46, 579.43, 563.40 (100), 536.39, 516.33, 492.32, 477.26, 314.61, 299.51	Isorhamnetin 3-*O*-rutinoside	624.16	C_28_H_32_O_16_
6	4.04	593.15	413.07, 314.64, 284.52, 276.68 (100), 240.36	Kaempferol 3-*O*-[2″-*O* (glycopyranoside)]-rhamnopyranoside	594.15	C_27_H_30_O_15_
7	4.1	593.20	475.21, 356.76, 326.65, 284.53 (100), 228.38	Kaempferol 3-*O*-rutinoside	594.15	C_27_H_30_O_15_
8	4.06	593.15	413.07, 314.64, 284.52, 276.68 (100), 240.36	Kaempferol 7-*O*-neohesperidoside	594.15	C_27_H_30_O_15_
9	4.10	594.16	284.46 (100), 226.53	Keracyanin	630.13	C_27_H_31_ClO_15_
10	6.24	755.44	593.47, 575.42 (100), 477.07, 431.07, 413.04, 276.58	Quercetin 3-*O*-[2″-*O*-(6″-*O*-*p*-coumaroyl)-*β*-D-glucopyranosyl]-*α*-L-rhamnopyranoside	756.19	C_36_H_36_O_18_
11	8.03	987.52	948.95, 729.61, 654.46, 431.01, 414.80 396.82 (100)	Soyasaponin B	942.51	C_48_H_78_O_18_
12	16.60	675.41	415.100 , 397.105 (100)	DGMG 18:3	676.36	C_33_H_56_O_14_
13	3.88	609.15	573.43, 561.42, 518.31, 501.27, 429.07, 300.54 (100), 292.68	Rutin	610.15	C_27_H_30_O_16_
14	4.66	712.40	550.63, 523.60 (100)	Soyacerebroside 1	713.54	C_40_H_75_NO_9_
15	3.75	755.21	709.90, 609.38, 593.46, 575.42 (100), 477.05, 431.07, 413.04, 276.58	Quercetin 3-*O*-[2″-*O*-(6'''-*O*-p-coumaroyl)-*β*-D-glucopyranosyl]-*α*-L-rhamnopyranoside	756.19	C_36_H_36_O_18_

*n*-Hexane fraction of *M. azedarach* leaves						

4∗	4.06	463.09	442.84, 432.77, 414.85, 342.58, 298.31(100)	Isoquercetin	464.09	C_21_H_20_O_12_
8∗	4.04	593.15	413.07, 314.64, 284.52, 276.68 (100), 240.36	Kaempferol 7-*O*-neohesperidoside	594.15	C_27_H_30_O_15_
14∗	4.66	712.40	550.63, 523.60 (100)	Soyacerebroside I	713.54	C_40_H_75_NO_9_
16	3.88	609.15	573.43, 561.42, 518.31, 501.27, 429.09, 300.54 (100), 292.68	Quercetin 3-*O*-neohesperidoside	610.15	C_27_H_30_O_16_
17	6.62	307.19	278.54, 262.57, 260.39, 198.318 (100), 124.00	Fatty acid 18:4	308.19	C_18_H_28_O_4_
18	4.21	559.31	397.044, 380.172, 378. 95, 350.967, 160.076, 158.104 (100)	MGMG 18:3	560.0	C_27_H_46_O_9_
19	6.97	721.36	466.39, 401.19, 326.81, 254.53 (100), 240.64	DGMG 18:3	676.797	C_33_H_56_O_14_
20	16.60	675.36	415.100, 397.105 (100)	DGMG 18:3	676.36	C_33_H_56_O_14_

Chloroform fraction of *M. azedarach* leaves						

8∗∗	4.04	593.15	413.07, 314.64, 284.52, 276.68 (100), 240.36	Kaempferol-7-neohesperidoside	594.15	C_27_H_30_O_15_
21	1.15	301.04	254.27 (100), 137.923, 136.81, 122.922	Quercetin	302.04	C_15_H_10_O_7_
22	6.13	697.32	515.079, 415.042 (100), 326.824, 278.54, 212.211	Momordicoside	696.40	C_37_H_60_O_12_
23	3.75	755.21	709.90, 609.38, 593.46, 575.42 (100), 477.05, 413.04, 431.07, 276.58	Quercetin 3-*O*-[2-*O*-6-z-p-coumaroyl-glucopyranoside]-rhamnopyranoside	756.19	C_36_H_36_O_18_
14∗∗	4.66	712.40	550.63, 523.60 (100)	Soyacerebroside I	713.54	C_40_H_75_NO_9_
9∗	4.10	594.16	284.46 (100), 226.53	Keracyanin	630.13	C_27_H_31_ClO_15_
24	4.61	593.19	549.42, 431.22, 366.813, 284.53 (100), 206.206, 168.208	Isosakuranetin-7-*O*-neohesperidoside	594.19	C_28_H_34_O_14_

Ethyl acetate fraction of *M. azedarach* leaves						

4∗∗	4.06	463.38	442.84, 432.77, 414.85, 342.58, 298.31(100)	Isoquercetin	464.09	C_21_H_20_O_12_
25	4.04	593.15	413.07, 314.64, 284.52, 276.68 (100), 240.36	Kaempferol 3-*O*-[2-*O*-(glucopyranoside)] rhamnopyranoside	594.15	C_27_H_30_O_15_

*n*-Butanol fraction of *M. azedarach* leaves						

26	3.84	739.21	559.43, 558.47, 430.97, 326.66, 284.47 (100)	Robinin	740.21	C_33_H_40_O_19_
27	3.81	625.14	462.08, 444.11, 358.90, 315.53 (100), 270.31	Isorhamnetin-3-*O*-galactoside-6''-rhamnoside	624.16	C_28_H_32_O_16_
28	4.1	593.20	475.21, 356.76, 326.65, 285.44, 276.68 (100), 228.38	Nicotiflorin	594.15	C_27_H_30_O_15_
15∗	3.73	755.18	609.387 (100), 489.173, 342.72, 300.56, 298.603, 270.505	Quercetin 3-*O*-[2''-*O*-(6'''-*O*-p-coumaroyl)-*β*-D-glucopyranosyl]-*α*-L-rhamnopyranoside	756.19	C_36_H_36_O_18_
13∗	3.88	609.15	573.43, 561.42, 518.31, 501.27, 429.07, 300.54 (100), 292.68	Rutoside (rutin)	610.15	C_27_H_30_O_16_
29	10.49	574.45	427.168, 349.22, 332.84 (100), 265.761, 246.24, 240.59	Sulfobacin B	575.45	C_32_H_65_NO_5_S

Aqueous fraction of *M. azedarach* leaves						

23∗	3.71	755.18	609.387 (100), 489.173, 342.72, 300.56, 298.603, 270.505	Quercetin 3-*O*-[2-*O*-6-z-p-coumaroyl-glucopyranoside]-rhamnopyranoside	756.7	C_36_H_36_O_18_
13∗∗	3.88	609.15	573.43, 561.42, 518.31, 501.27, 429.07, 300.54 (100), 292.68	Rutin	610.5	C_27_H_30_*O*_16_

RETRACTED

## Data Availability

The data will be available on demand.
